The article "Long non-coding RNA LBX2-AS1 enhances glioma proliferation through downregulating microRNA-491-5p" was retracted in 2020. Reasons: errors in the analysis; errors in the methods; errors in the results or conclusions.

# Long non-coding RNA LBX2-AS1 enhances glioma proliferation through downregulating microRNA-491-5p

**DOI:** 10.1186/s12935-020-01433-2

**Published:** 2020-08-26

**Authors:** Qunbang Chen, Jian Gao, Yingjia Zhao, Ruizhe Hou

**Affiliations:** 1 Department of Neurosurgery, China-Japan Union Hospital of Jilin University, Changchun, 130033 Jilin China; 2 Department of Gynecology and Obstetric, The Second Hospital of Jilin University, Changchun, 130000 Jilin China

**Keywords:** LBX2-AS1, miR-491-5p, Cell proliferation, Cell apoptosis, Glioma, TRIM28

## Abstract

**Background:**

Dysregulation of lncRNAs is frequent in glioma and has emerged as an important mechanism involved in tumorigenesis. Previous analysis of Chinese Glioma Genome Atlas (CGGA) database indicated that LBX2-AS1 expression is one of differentially expression lncRNA between lower grade glioma (LGG) (grade II and III) and glioblastoma multiforme (GBM). However, the function and mechanism of LBX2-AS1 in glioma has not been evaluated yet.

**Methods:**

Here, we analyzed the expression of LBX2-AS1 in GTEx data (normal brain), TCGA-LGG and TCGA-GBM. RT-PCR was performed to detect LBX2-AS1 in surgery obtained normal brain and glioma. CCK-8 kit and Annexin V-FITC-PI Apoptosis Detection Kit were used to study the function of LBX2-AS1 on glioma proliferation and apoptosis. Bioinformatic analysis, RNA immunoprecipitation, RT-PCR, western blotting and dual luciferase reporter assay were carried out to investigate the target miRNA of LBX2-AS1. The discovered mechanism was validated by the rescue assay.

**Results:**

Following study of GTEx and TCGA data, LBX2-AS1 was significantly elevated in glioma compared with normal brain and in GBM compared with LGG. Higher expression of LBX2-AS1 was associated with poor prognosis of patients with glioma. Expression of LBX2-AS1 was positively correlated with pathology classification of glioma. Knockdown of LBX2-AS1 inhibited cell proliferation and induced cell apoptosis in glioma. LBX2-AS1 have complimentary binding site for tumor suppressor miR-491-5p and we showed that LBX2-AS1 sponged miR-491-5p to upregulate TRIM28 expression in glioma cells. TRIM28 overexpression attenuated the effect of LBX2-AS1 knockdown on glioma cells.

**Conclusions:**

In conclusion, LBX2-AS1 was an increased lncRNA in glioma. Mechanistically, LBX2-AS1 promoted glioma cell proliferation and resistance to cell apoptosis via sponging miR-491-5p.

## Background

Gliomas are the most common primary cancer types derived from the neural ectoderm, accounting for approximately half of all brain malignancy [1]. Gliomas are histologic classified into several groups including grade II oligodendrogliomas and astrocytomas, and grade III anaplastic oligodendrogliomas, anaplastic astrocytomas, anaplastic oligoastrocytomas, anaplastic ependymomas, and grade IV glioblastomas (GBM) according to World Health Organization (WHO) classification [2, 3]. Overall, gliomas are lethal cancer type and patients with high grade glioma (GBM) have a median overall survival less than one year [4]. The worse prognosis of patients with glioma is partly due to resistance to radiotherapy and chemotherapy induced cell apoptosis and the strong proliferation ability of cancer cells [5, 6].

The article "Long non-coding RNA LBX2-AS1 enhances glioma proliferation through downregulating microRNA-491-5p" was retracted in 2020. Reasons: errors in the analysis; errors in the methods; errors in the results or conclusions.

Long non-coding RNAs are RNA molecules longer than 200 nucleotides without protein coding potential [7]. As part of competing endogenous RNA (ceRNA) network, the function of many lncRNAs rely on their interaction with microRNAs (miRNAs) to regulate expression of gene with same miRNA response elements (MREs) [8]. Accumulating evidences suggested that lncRNAs are implicated in glioma progression via sponging miRNAs [9–11]. For example, lncRNA CCAT1 sponged miR-181b, increased miR-181b target FGFR3 and PDGFRα and promoted glioma cell proliferation, invasion and resistance to cell apoptosis [12]. LBX2-AS1 is a recently identified cancer associated lncRNA in several cancer types [13]. Overexpression of LBX2-AS1 has been reported in hepatocellular carcinoma, gastric cancer, non-small cell lung cancer and esophageal squamous cell carcinoma and it promoted cancer cell proliferation with different mechanism in different cell background [13–16]. In non-small cell lung cancer, LBX2-AS1 activated Notch pathway to facilitate cancer cell proliferation, migration and invasion [13]. In esophageal squamous cell carcinoma, LBX2-AS1 stabilized ZEB1 and ZEB2 to promote epithelial-mesenchymal transition of cancer cells [16]. LBX2-AS1 is one of 169 aberrantly expressed lncRNAs between LGG and GBM from CGGA database [17]. The biological role of LBX2-AS1 has not been examined in glioma.

The current study revealed that LBX2-AS1 was a significantly upregulated lncRNA in glioma and its expression associated with prognosis of patients with glioma. We aimed to explore the biological role and molecular mechanism of LBX2-AS1 in glioma.

## Materials and methods

### Patients and samples

Tissue samples, including 9 normal brains and 51 glioma tissues were obtained from the therapeutic surgery of patients in the Third Hospital of Jilin University during June 2016 to July 2019. Samples were confirmed histologically by two neuropathologists following the criteria of 2007 WHO classification guidelines. Written informed consents were provided and the protocol was approved by the Third Hospital of Jilin University institutional review board. The collected samples were stored at -80℃ until RNA extraction.

The article "Long non-coding RNA LBX2-AS1 enhances glioma proliferation through downregulating microRNA-491-5p" was retracted in 2020. Reasons: errors in the analysis; errors in the methods; errors in the results or conclusions.

### Cell lines and culture

Human glioma cell lines U87MG, U251MG and A172 were purchased from ATCC (Manassas, VA). Human astrocyte cell line (NHA) was bought from the Cell Bank of the Chinese Academy of Sciences (Shanghai, China). Cells were maintained in Dulbecco’s Modified Eagle Medium (Invitrogen, Carlsbad, CA) supplemented with 10% FBS (Gibco, Rockville, MD). All cells were cultured in a humid incubator with 5% CO_2_ at 37℃.

### RNA immunoprecipitation (RIP) assay

A Magna RIP RNA-Binding Protein Immunoprecipitation kit (Millipore, Bedford, MA) was used to perform RIP. In a brief, U87MG cell lysate was incubated with magnetic beads pre-incubated with mouse IgG (negative control) or human anti-Ago2 antibody (Cat. no. 04-642, Millipore, Billerica, MA). Total RNAs were then isolated by TRIzol reagent and detected by RT-PCR to measure the enrichment of miR-491-5p and LBX2-AS1.

### Bioinformatic analysis

The expression of LBX2-AS1 in GTEx, TCGA-LGG and TCGA-GBM projects were obtained from GEPIA software (http://gepia.cancer-pku.cn/) which was also used to study the association between LBX2-AS1 expression and prognosis of patients with glioma. The association between LBX2-AS1 and TRIM28 was also analyzed by GEPIA based on TCGA-LGG project. ENCORI software (http://starbase.sysu.edu.cn/) was used to predict target miRNAs of LBX2-AS1 and the association between LBX2-AS1 and miR-491-5p expression in TCGA-LGG.

### Quantitative real-time polymerase chain reaction

Total RNA was extracted from cells and tissues with TRIzol reagent (Invitrogen). RNA concentration was detected by NanoDrop 2000 (Thermo Fisher Scientific, Wilmington, DE). First-stranded cDNA was synthesized from RNA with Prime-Script RT Reagent Kit (TaKaRa, Dalian, China). Real-time polymerase chain reaction was performed with SYBR Prime Script RT‐PCR kit (TaKaRa) on an ABI 7500 Fast Real‐Time PCR system (Applied Biosystems, Foster City, CA). mRNA and lncRNA were normalized to β-actin. miRNA was normalized to U6. The relative expression of gene was calculated by 2^−ΔΔCt^ method. Primer sequences were listed in Table 1.

**Table 1:** Sequence of RT-qPCR primers

Primer		Sequence
LBX2-AS1	Forward	5′-AATTCGCAGGAAGGGGAGTG-3′
	Reverse	5'-TGCCAAACCTGGGACAAACT-3′
TRIM28	Forward	5'-TGAGACCTGTGTAGAGGCG-3′
	Reverse	5′-CGTTCACCATCCCGAGACTT-3′
β-actin	Forward	5′-CATGTACGTTGCTATCCAGGC-3′
	Reverse	5′-CTCCTTAATGTCACGCACGAT-3′
miR-491-5p	Stem loop	5′-CTCAACTGGTGTCGTGGAGTCGGCAATTCAGTTGAGCCTCAT-3′
	Forward	5′-TCGGCAGGAGTGGGGAACCCTTC-3′
	Reverse	5′-CTCAACTGGTGTCGTGGA-3′
U6 snRNA	Stem loop	5′-CGCTTCACGAATTTGCGTGTCA-3′
	Forward	5′-GCTTCGGCAGCACATATACTAAAAT-3′
	Reverse	5′-CGCTTCACGAATTTGCGTGTCAT-3′

The article "Long non-coding RNA LBX2-AS1 enhances glioma proliferation through downregulating microRNA-491-5p" was retracted in 2020. Reasons: errors in the analysis; errors in the methods; errors in the results or conclusions.

### Cell transfection

si-Control (5′-UUCUCCGAACGUGUCACGUTT-3′), si-LBX2-AS1-1 (5′-CCAUUAAUUCAGCAAACAUUCCUTT-3') and si-LBX2-AS1-2 (5′-UGAUUUUUUAAAGAAAAAUCCAATT-3′) were designed and synthesized by GenePharma (Suzhou, China). For transfection, siRNA was mixed with Lipofectamine RNAiMax (Invitrogen) in serum-free DMEM and added into cultured cells. miR-NC (5′-CAGCUGGUUGAAGGGGACCAAA-3′), miR-491-5p mimic (5′-AGUGGGGAACCCUUCCAUGAGG-3′) and miR-491-5p inhibitor (5′-CCUCAUGGAAGGGUUCCCCACU-3′) was synthesized by RiBo Bio (Guangzhou, China). These miR-NC, miR-491-5p mimic and inhibitor was mixed with Lipofectamine 3000 (Invitrogen) in serum-free DMEM and added into cultured cells. The transfection efficiency was detected 48 h after transfection.

### Western blotting

p-S6K (Cat. 9208) and S6K (Cat. 9202) antibodies were obtained from CST (Beverly, CA). TRIM28 antibody (Cat. 61,174) was product of Active Motif (Carlsbad, CA). β-actin antibody (Cat. KC-5A08) was bought from Aksomics (Shanghai, China). HRP-conjugated mouse (Cat. ab6728) and rabbit (Cat. ab6721) antibodies were purchased from Abcam (Cambridge, UK). RIPA lysis buffer (Thermo Fisher Scientific) was used to extract proteins from cells. Proteins were separated by an SDS-PAGE gel and transferred to PVDF membranes. The membrane was blocked in 5% non-fat milk and incubated with primary and secondary antibody. ECL Substrate (Thermo Fisher Scientific) was used to develop blots.

### Cell proliferation and apoptosis assay

The CCK-8 kit (Beyotime, Shanghai, China) was used to detect cell proliferative ability. Briefly, 10 µL CCK-8 was mixed with culture medium and sustained for an additional 2 h. After that, the absorbance at 450 nm of each well was detected by a Microplate Reader (Bio-Rad, Hercules, CA). Percentage of apoptotic cells was measured with Dead Cell Apoptosis Kit with Annexin V FITC and PI kit (Invitrogen) by flow cytometry analysis. Cells were suspended in Annexin-V binding buffer provided by the kit and stained with Annexin-V FITC and PI sequentially. The cells were then subjected to flow cytometry analysis. Cells positive for Annexin V with or without PI positive were apoptotic cells.

### Dual luciferase reporter assay

LBX2-AS1, TRIM28 3′UTR or their mutant forms were inserted into pmirGLO luciferase vector. These vectors were then co-transfected with miR-NC or miR-491-5p into cells by Lipofectamine 3000. After 48 h, the relative luciferase activity of each group was measured with the Dual Luciferase Reporter Assay System kit (Promega Corp., Madison, WI). Firefly luciferase was normalized to Renilla luciferase.

The article "Long non-coding RNA LBX2-AS1 enhances glioma proliferation through downregulating microRNA-491-5p" was retracted in 2020. Reasons: errors in the analysis; errors in the methods; errors in the results or conclusions.

### Bioinformatic analysis

The data were analyzed with Graphpad Prism 6.0 software. The difference between the groups were examined with Student’s t test or one-way ANOVA analysis followed by Tukey test. The association between expression of two genes was studied with Pearson correlation analysis. P value less than 0.05 was considered as statistically significant.

## Results

### LBX2-AS1 was overexpressed in glioma and its expression was associated with poor prognosis of glioma patients

We firstly studied the expression of LBX2-AS1 in normal brains from GTEx project, low grade glioma (LGG) and glioblastoma (GBM) from TCGA project. The results suggested that LBX2-AS1 was 4-fold and 10-fold highly expressed in glioma tissues from TCGA-LGG and TCGA-GBM compared with normal brains from GTEx, expression of LBX2-AS1 was nearly 3-fold higher in high-grade glioma (GBM) compared with low-grade glioma (LGG) (Fig. 1a). We collected 9 normal brains and 51 glioma tissues and analyzed LBX2-AS1 expression by RT-PCR. It showed that LBX2-AS1 was approximately 3-fold highly expressed in glioma compared with normal brains (Fig. 1b). Furthermore, LBX2-AS1 was increased in high grade glioma (Grade IV vs. Grade III, Grade III vs. Grade II) (Fig. 1c). Retrospective analysis of the clinical outcome from TCGA-LGG and TCGA-GBM datasets suggested that LBX2-AS1 high expression group (n = 337) have a shorter disease-free survival compared with LBX2-AS1 low expression group (n = 335) (Fig. 1d). Meanwhile, patients with higher expression of LBX2-AS1 showed a shorter overall survival time compared with their counterparts (Fig. 1e).

**Fig. 1:** LBX2-AS1 was an upregulated lncRNA in glioma.** a** Analysis of LBX2-AS1 expression in normal brains from GTEx project and glioma tissues from TCGA-LGG and TCGA-GBM projects. **b** RT-PCR detection of LBX2-AS1 expression in normal brains and gliomas. **c** Comparison of LBX2-AS1 expression in normal brain, grade II glioma, grade III glioma and grade IV glioma. **d**, **e** Kaplan Meier-plotter analysis of association between LBX2-AS1 expression and disease-free survival **d**, overall survival **e** of patients with glioma from TCGA-LGG and TCGA-GBM projects. ***, p < 0.001

### LBX2-AS1 was negatively associated with miR-491-5p in glioma

To study the mechanism of LBX2-AS1 in glioma, we firstly used RT-PCR method to detect LBX2-AS1 expression in a panel of glioma cell lines. Expression of LBX2-AS1 was significantly increased in U87MG, U251MG and A172 cells in comparison with normal human astrocyte (NHA) (Fig. 2a). LBX2-AS1 functioned as a ceRNA to exert its function on cell behavior [15]. We used the following method to screen for target miRNAs of LBX2-AS1 (Fig. 2b). Firstly, ENCORI database prediction showed that LBX2-AS1 have 28 putative binding sites for 27 miRNAs. Pearson correlation analysis suggested that the expression of three of these miRNAs (miR-1911-5p, miR-219a-2-3p and miR-491-5p) were negatively correlated with LBX2-AS1 expression in TCGA-LGG dataset. In these three miRNAs, miR-491-5p was an upregulated miRNA in TCGA data of glioma as reported by Qi et al. [18]. The strong negative correlation between miR-491-5p and LBX2-AS1 expression was showed in Fig. 2c (Pearson r = − 0.383, p < 0.001). Expression of miR-491-5p was decreased by more than 40% in collected glioma compared with normal brains (Fig. 2d). In contrast to LBX2-AS1, miR-491-5p was lowly expressed in high grade glioma compared with those of low grade (Grade IV vs. Grade III) (Fig. 2e). The negative correlation between LBX2-AS1 and miR-491-5p expression was also observed in these glioma tissues (Fig. 2f). To study whether LBX2-AS1 interact with miR-491-5p, we firstly transfected miR-491-5p mimic into U87MG and U251MG cells to elevate miR-491-5p expression (Fig. 2g). Full length of LBX2-AS1 was inserted into luciferase vector pmirGLO. Luciferase reporter assay showed that miR-491-5p overexpression did repress luciferase activity of pmirGLO-LBX2-AS1 by around half in U87MG (Fig. 2h) and U251MG cells (Fig. 2i). More importantly, RIP assay showed that Ago2 antibody enriched both LBX2-AS1 and miR-491-5p in U87MG cells (Fig. 2j). These data implied that LBX2-AS1 might regulate miR-491-5p in glioma cells.

The article "Long non-coding RNA LBX2-AS1 enhances glioma proliferation through downregulating microRNA-491-5p" was retracted in 2020. Reasons: errors in the analysis; errors in the methods; errors in the results or conclusions.

**Fig. 2:** LBX2-AS1 expression was associated with miR-491-5p levels in glioma. **a** RT-PCR detection of LBX2-AS1 expression in a panel of glioma cell lines U87MG, U251MG, A172 and normal human astrocyte (NHA). **b** Flow chart of screen for target miRNAs of LBX2-AS1 in glioma. **c** The association between LBX2-AS1 and miR-491-5p expression in TCGA-LGG project was analyzed by Pearson correlation analysis. **d** RT-PCR detection of miR-491-5p expression in normal brains and gliomas. **e** Comparison of miR-491-5p expression in normal brain, grade II glioma, grade III glioma and grade IV glioma. **f** The association between LBX2-AS1 and miR-491-5p expression in collected glioma samples was analyzed by Pearson correlation analysis. **g** The expression of miR-491-5p was detected in U87MG and U251MG cells transfected with miR-NC or miR-491-5p mimic. In U87MG (**h**) and U251MG (**i**) cells, the luciferase activity of pmirGLO (empty vector as the control group) and pmirGLO-LBX2-AS1 was detected. J. RIP assay was performed with IgG and Ago2 antibody, followed by RT-PCR detection of LBX2-AS1 and miR-491-5p levels. *, p < 0.05; ***, p < 0.001

The article "Long non-coding RNA LBX2-AS1 enhances glioma proliferation through downregulating microRNA-491-5p" was retracted in 2020. Reasons: errors in the analysis; errors in the methods; errors in the results or conclusions.

### A mutual regulatory association between miR-491-5p and LBX2-AS1 in glioma

To study the association between miR-491-5p and LBX2-AS1, we transfected increasing concentrations (50 nM and 100 nM) of miR-491-5p mimic into U87MG and U251MG cells. Expression of miR-491-5p was increased by 5 and 9-fold in U87MG cells transfected with 50 nM and 100 nM miR-491-5p mimic respectively (Fig. 3a). In U251MG cells, miR-491-5p levels were increased by 3.5 and 4.5-fold after transfection of 50 nM and 100 nM miR-491-5p (Fig. 3a). Overexpression of miR-491-5p decreased LBX2-AS1 expression by more than half in U87MG and U251MG cells and lower expression of LBX2-AS1 was observed in cells with high concentration of miR-491-5p mimic (Fig. 3b). Two independent siRNAs targeting LBX2-AS1 (si-LBX2-AS1-1 and si-LBX2-AS1-2) were transfected into glioma cells. These siRNAs greatly decreased LBX2-AS1 expression by more than 70% in U87MG and U251MG cells (Fig. 3c). In addition, knockdown of LBX2-AS1 increased miR-491-5p expression in U87MG and U251MG cells (Fig. 3d). Transfection of si-LBX2-AS1-2, which reduced LBX2-AS1 expression in a relatively larger extent compared with si-LBX2-AS1-1, was more effective in upregulation of miR-491-5p expression in the cells (Fig. 3d), indicating the negative regulation of miR-491-5p by LBX2-AS1. We analyzed the complementary site between LBX2-AS1 and miR-491-5p and constructed pmirGLO vector with mutant LBX2-AS1 (LBX2-AS1 Mut) (Fig. 3e). Overexpression of miR-491-5p repressed luciferase activity of LBX2-AS1 WT instead of LBX2-AS1 Mut in U87MG (Fig. 3f) and U251MG cells (Fig. 3g).

**Fig. 3:** miR-491-5p mutually regulated LBX2-AS1 in glioma. miR-491-5p (**a**) and LBX2-AS1 (**b**) expression was detected in U87MG and U251MG cells transfected with miR-NC or increasing concentration of miR-491-5p mimic (50 nM, 100 nM). **c** LBX2-AS1 expression was detected in U87MG and U251MG cells transfected with si-Control or si-LBX2-AS1-1 or si-LBX2-AS1-2 by RT-PCR. **d** mir-491-5p expression was detected in U87MG and U251MG cells transfected with si-Control or si-LBX2-AS1-1 or si-LBX2-AS1-2. **e** Sequence alignment of LBX2-AS1 WT, LBX2-AS1 Mut and miR-491-5p. Luciferase activity was detected in U87MG (**f**) and U251MG (**g**) cells transfected with LBX2-AS1 WT or LBX2-AS1 Mut. **, p < 0.01; ***, p < 0.001

### LBX2-AS1 upregulated TRIM28 expression in glioma

Previous study suggested that miR-491-5p targeted TRIM28 to regulate glioma cell proliferation [18]. After investigation of TRIM28 and LBX2-AS1 expression in TCGA-LGG and TCGA-GBM datasets, it was found that TRIM28 was positively correlated with LBX2-AS1 expression in glioma (Pearson r = 0.300, p < 0.001) (Fig. 4a). Additionally, TRIM28 was highly expressed in our collected glioma samples compared with normal brains (Fig. 4b). Pearson correlation analysis showed a strong positive correlation between LBX2-AS1 and TRIM28 levels in our collected glioma tissues (Pearson r = 0.623, p < 0.001) (Fig. 4c). Knockdown of LBX2-AS1 decreased approximately 50% TRIM28 mRNA expression in U87MG and U251MG cells (Fig. 4d). TRIM28 induced dephosphorylation of S6K to control glioma development [19]. LBX2-AS1 downregulation decreased TRIM28 protein expression and the downstream phosphorylation of S6K (p-S6K) by half in U87MG cells as measured by western blotting (Fig. 4e). Similarly, LBX2-AS1 knockdown also decreased TRIM28 and p-S6K in U251MG cells to the same extent as in U87MG (Fig. 4f).

The article "Long non-coding RNA LBX2-AS1 enhances glioma proliferation through downregulating microRNA-491-5p" was retracted in 2020. Reasons: errors in the analysis; errors in the methods; errors in the results or conclusions.

**Fig. 4:** LBX2-AS1 regulated TRIM28 expression in glioma.** a** Pearson correlation analysis of LBX2-AS1 and TRIM28 expression in TCGA-LGG and TCGA-GBM projects. **b** RT-PCR detection of TRIM28 mRNA expression in normal brains and gliomas. **c** Pearson correlation analysis of LBX2-AS1 and TRIM28 expression in collected glioma. **d** TRIM28 mRNA expression was detected in U87MG and U251MG cells transfected with si-Control or si-LBX2-AS1-1 or si-LBX2-AS1-2 by RT-PCR. TRIM28, p-S6K protein expression was detected in U87MG (**e**) and U251MG (**f**) cells transfected with si-Control or si-LBX2-AS1-1 or si-LBX2-AS1-2 by western blotting. Β-actin and S6K were internal controls for TRIM28 and p-S6K. **, p < 0.01; ***, p < 0.001

### LBX2-AS1 regulated TRIM28 via sponging miR-491-5p

We first transfected miR-491-5p inhibitor into U87MG and U251MG cells to decrease miR-491-5p expression in these cells, miR-491-5p inhibitor decreased 70% miR-491-5p expression in cells (Fig. 5a). We found that miR-491-5p inhibitor could reverse the downregulation of TRIM28 mRNA expression by si-LBX2-AS1-1 in U87MG and U251MG cells (Fig. 5b). Western blotting further showed that miR-491-5p inhibitor could reverse the downregulation of TRIM28 protein expression by si-LBX2-AS1-1 in U87MG and U251MG cells (Fig. 5c). Luciferase vectors containing wild-type and mutant TRIM28 3′UTR (TRIM28 3′UTR WT, TRIM28 3′UTR Mut) were constructed (Fig. 5d). In U87MG cells, miR-491-5p inhibitor could reverse the repression of luciferase activity of TRIM28 3′UTR WT by si-LBX2-AS1-1 (Fig. 5e). These data collectively demonstrated a LBX2-AS1/miR-491-5p/TRIM28 axis in glioma.

**Fig. 5:** LBX2-AS1 regulated TRIM28 expression via sponging miR-491-5p. **a** The expression of miR-491-5p was detected in U87MG and U251MG cells transfected with miR-NC or miR-491-5p inhibitor. **b** The expression of TRIM28 mRNA was detected in U87MG and U251MG cells transfected with miR-NC or miR-491-5p inhibitor in combination with si-Control or si-LBX2-AS1-1 by RT-PCR. **c** The expression of TRIM28 protein was detected in U87MG cells transfected with miR-NC or miR-491-5p inhibitor in combination with si-Control or si-LBX2-AS1-1 by western blotting. **d** Sequence alignment of LBX2-AS1 TRIM28 3′UTR WT, TRIM28 3′UTR Mut and miR-491-5p. **e** Luciferase activity was detected in U87MG cells transfected with TRIM28 3′UTR WT or TRIM28 3′UTR Mut in combination with si-Control or si-LBX2-AS1-1 and miR-NC or miR-491-5p inhibitor. **, p < 0.01; ***, p < 0.001

The article "Long non-coding RNA LBX2-AS1 enhances glioma proliferation through downregulating microRNA-491-5p" was retracted in 2020. Reasons: errors in the analysis; errors in the methods; errors in the results or conclusions.

### **LBX2-AS1 promoted cell proliferation and resistance to cell apoptosis by repression of miR-491-5p**

.

It is known that aberrant expression of miR-491-5p and TRIM28 mediated glioma cell proliferation and survival [18]. To investigate the impact of the LBX2-AS1/miR-491-5p/TRIM28 axis on cell proliferation, we performed CCK-8 assay in glioma cells transfected with si-LBX2-AS1 with or without miR-491-5p inhibitor. Knockdown of LBX2-AS1 inhibited cell proliferation in U87MG cells and the effect of si-LBX2-AS1 was reversed upon co-transfection of miR-491-5p inhibitor (Fig. 6a). In consistent with U87MG, si-LBX2-AS1-1 and si-LBX2-AS1-2 inhibited U251MG cell proliferation which was attenuated by miR-491-5p inhibitor (Fig. 6b). With the flow cytometry, we also found that LBX2-AS1 knockdown induced cell apoptosis in U87MG cells and the effect of si-LBX2-AS1 was partially rescued by miR-491-5p inhibitor (Fig. 6c). Similar results were found in U251MG cells (Fig. 6d). These data manifested that LBX2-AS1 mainly relied on regulation of miR-491-5p to mediate glioma cell proliferation and survival.

**Fig. 6:** LBX2-AS1 regulated cell proliferation and apoptosis via sponging miR-491-5p. Transfection of si-LBX2-AS1-1 or si-LBX2-AS1-2 inhibited cell proliferation and was reversed by transfection of miR-491-5p inhibitor in U87MG (**a**) and U251MG (**b**) cells as indicated by CCK-8 assay. Transfection of si-LBX2-AS1-1 or si-LBX2-AS1-2 induced cell apoptosis and was partially reversed by transfection of miR-491-5p inhibitor in U87MG (**c**) and U251MG (**d**) cells as indicated by flow cytometry analysis. **, p < 0.01; ***, p < 0.001

## Discussion

LBX2-AS1 is a most recently identified oncogenic lncRNA across several cancer types. LBX2-AS1 was reported as a highly expressed lncRNA in non-small cell lung cancer, especially in tumors of advanced stage [13]. High expression of LBX2-AS1 was also found in stomach adenocarcinoma and hepatocellular carcinoma [14, 15]. Here, we analyzed LBX2-AS1 expression in glioma by using data of TCGA-LGG and TCGA-GBM projects in combination with normal brains from GTEx project. Similar to observation in other cancer types, it was observed that LBX2-AS1 was increased in glioma especially high-grade glioma (GBM). We further revealed that patients with high expression of LBX2-AS1 have a short disease-free survival and overall survival, indicating LBX2-AS1 could predict poor prognosis of glioma. As the published studies showed that LBX2-AS1 was associated with poor prognosis of patients with hepatocellular carcinoma and non-small cell lung cancer [13, 14], the findings suggested that LBX2-AS1 might be a predictive biomark for a variety of cancer types.

The article "Long non-coding RNA LBX2-AS1 enhances glioma proliferation through downregulating microRNA-491-5p" was retracted in 2020. Reasons: errors in the analysis; errors in the methods; errors in the results or conclusions.

LBX2-AS1 exerted its pro-cancer functions via acting as a ceRNA to sponge tumor suppressive miRNAs. For example, LBX2-AS1 directly interacted with tumor suppressive miR-384 to enhance cell proliferation and resistance to cell apoptosis in hepatocellular carcinoma [14]. Our bioinformatic analysis indicated that LBX2-AS1 have a putative binding site for miR-491-5p. miR-491-5p was a tumor suppressor in several cancer types [20–23]. Aberrant expression of miR-491-5p was the consequence of upregulated circRNA circ_0001361 and lncRNA XIST in bladder cancer and nasopharyngeal carcinoma respectively [24, 25]. In glioma, miR-491-5p was decreased in cancer tissues and correlated with good prognosis [18]. We confirmed miR-491-5p as a target miRNA of LBX2-AS1 in glioma. Upregulation of miR-491-5p induced cancer cell apoptosis to cease cell proliferation [26, 27]. We showed that LBX2-AS1 mediated glioma cell proliferation and resistance to cell apoptosis, downregulation of miR-491-5p could partially rescue the impact of LBX2-AS1 knockdown on glioma cell proliferation and apoptosis. Thus, the current data indicated a novel interaction between LBX2-AS1 and miR-491-5p and manifested that LBX2-AS1 promoted glioma proliferation via sponging miR-491-5p. However, as the cell apoptosis induced by LBX2-AS1 knockdown was not fully rescued by miR-491-5p downregulation, we believe there are several other mechanisms underlying the function of LBX2-AS1 in glioma. For example, the Notch signaling was regulated by LBX2-AS1 in non-small cell lung cancer and the activity of Notch signaling determined the cell apoptosis in glioma [13, 28]. It remains unknown whether LXB2-AS1 uses the same mechanism to control Notch signaling in glioma. Future study will reveal the complexity of signaling network regulated by LBX2-AS1 in glioma. In addition, due to the involvement of miR-491-5p in cancer cell metastasis [21], further studies will be needed to evaluate the effect of LBX2-AS1 on glioma metastasis.

TRIM28 is a cancer-associated E3 ligase in several cancer types [29]. Upregulation of TRIM28 was found in glioma and the pro-proliferative function of TRIM28 was supported by *in vitro* and *in vivo* data [18, 19]. In glioma, TRIM28 mediated degradation of tumor suppressor AMPK, activated mTORC1 and regulated cell apoptosis [19]. TRIM28 expression was repressed by several non-coding RNA in different cell background [18, 30]. In the current study, in addition to the known miR-491-5p/TRIM28 interaction in glioma, we further discovered that lncRNA LBX2-AS1 could regulated TRIM28 via sponging miR-491-5p in glioma background. Mechanistically, TRIM28 form complex with MAGE to regulate mTOR activity and the downstream phosphorylation of S6K [19, 31, 32]. We found that LBX2-AS1 not only upregulated TRIM28 expression but also increased phosphorylation level of S6K in glioma cells. Therefore, the data revealed a LBX2-AS1/miR-491-5p/TRIM28 axis in glioma.

The article "Long non-coding RNA LBX2-AS1 enhances glioma proliferation through downregulating microRNA-491-5p" was retracted in 2020. Reasons: errors in the analysis; errors in the methods; errors in the results or conclusions.

## Conclusions

Our results suggested that lncRNA LBX2-AS1 promoted glioma cell proliferation and resistance to cell apoptosis via sponging miR-491-5p. LBX2-AS1 could be a novel biomarker for patients with glioma.

## Data Availability

All data generated or analyzed during this study are included in this published article.
